# A Real-Time Medical Ventilation on Heart Failure Analysis Based on Sleep Apnea Snore and Meta-Analysis

This article has been retracted.

**DOI:** 10.1155/2022/9979413

**Published:** 2022-04-11

**Authors:** Xin Liu, Yingxin Zhao

**Affiliations:** ^1^Department of Cardiology, Beijing Institute of Heart Lung and Blood Vessel Disease, Beijing Anzhen Hospital, Capital Medical University, Beijing 10002 Beijing, China; ^2^Cardiovascular Center, Beijing Tongren Hospital, Capital Medical University, Beijing 100176 Beijing, China

## Abstract

An issue with cardiac ventilation can result in death at any moment throughout a person's life. The apnea-hypopnea index (AHI) has historically been influenced by medical ventilation on heart failure; nevertheless, the sleep snore analysis is the best model to diagnose. The problems with ventilation are caused by problems with air pressure and blood circulation in the heart valves, where the pathological measures are continually detecting ventilation issues. Understanding the pathophysiology of OSA will have a direct impact on clinical treatment choices as well as the design of clinical studies. Treatments could be tailored to each patient's unique needs based on the fundamental reason to their OSA. Through the OSA treatment, patients could feel better, and understanding OSA symptoms and also outcomes will improve patient's health; as a result, the study reveals that most of the population are likely to benefit from specific OSA treatment approaches. For achieving the benefits of OSA treatment the classification accuracy is needed to be improved. So, in this research work, an LeNet-100 CNN-based deep learning technology is used to get information and apply the classification approaches. We obtained the heart failure dataset from the Kaggle website for conducting a meta-analysis. An accuracy of 93.25%, sensitivity of 97.29%, recall of 96.34%, and F measure of 95.34% had been attained. This approach outperforms the technology and is comparable to the present heart failure meta-analysis..

## 1. Introduction

The apnea-hypopnea index (AHI) has traditionally described the existence and state of the OSA (Obstructive Sleep Apnea). Despite its poor adherence rate, positive airway pressure continuation remains the healing of option because it consistently lowers the AHI when administered, while the response to alternative approaches is unpredictable. As a result, there is an increasing understanding that the AHI does not adequately identify the underlying cause (i.e., endotype) and clinical presentation of OSA in a person. OSA subtypes are defined and reviewed, as is the potential application of genetics in further refining illness categorization. We have made significant progress in identifying and evaluating physiological causes (or endotypes). Patients with OSA have frequent episodes of hypoxia and awakenings due to the obstruction of their upper airway during sleep. High sympathetic activity, frequent oxygen desaturations, and sleep fragmentation have been related to cardiovascular (such as high blood pressure, strokes, or myocardial infarction), metabolic (such as diabetes), and neurocognitive repercussions. Since the older population and the overweight pandemic are known to contribute to OSA risk, the prevalence of clinically significant OSA has been estimated to be over 10% of Americans (almost 13% of middle-aged men and 6% of American women). The frequency of Alzheimer's disease may be significantly greater among the elderly people.

Through these efforts, we have consistently identified three main subgroups defined by (1) interrupted sleep (i.e., insomnia) symptoms, (2) a relative absence of typical OSA symptoms, or (3) notable excessive daytime sleepiness. Beyond this, investigations in the Sleep Apnea Global Interdisciplinary Consortium (SAGIC), a globally ethnically diversified sample of individuals with OSA from sleep clinics, discovered two further subgroups defined by either upper airway symptoms or moderate sleepiness. Ultimately, the regularity of these outcomes provides strong evidence that clinical symptom categories represent real underlying disease traits. To appreciate the therapeutic value of SA symptom subgroups, it is vital to validate their link with meaningful outcomes. Toward this end, recent studies within the Icelandic Sleep Apnea Cohort (ISAC) demonstrated that symptom subtypes benefit in distinct ways with respect to symptom improvements after 2 years of treatment with continuous positive airway pressure (CPAP). Currently, however, it is questionable whether these symptom categories have different long-term health repercussions, particularly with regard to cardiovascular disease (CVD) (Figure 1).

Before looking at whether various subtypes are linked with a higher incidence of cardiovascular disease at baseline and a higher risk for cardiovascular outcomes over the follow-up period, we first validate the presence of comparable subtypes (AHI, 5).

The contribution of the paper is as follows:

- To obtain the information and apply the classification approaches by using deep learning technology called LeNet-100 CNN
- To compare the performance of LeNet-100 CNN classification technique with deep stacked and AGWO

## 2. Literature Survey

Edwards et al. show treatments could be tailored to each patient's unique needs based on the fundamental reason under OSA patients; Through the OSA treatment patients could feel better and understanding OSA symptoms and also outcomes will improve patient's health; as a result study reveal that most of the population likely to benefit from specific OSA treatment approaches [1]. Coleman et al. studied a treatment plan and evaluation algorithm for use into medical practice are presented. However, a complete evidence-based approach to this potentially effective medication is limited due to the absence of crucial clinical research [2]. Kersin et al. studied that automated tongue base excision and uvulopharyngoplasty improve respiratory function measurements. For individuals with OSAS, surgical treatment is as favorable to respiratory function as CPAP [3]. Carter describes that when fresh data are gathered for this research, they may be utilized in the public health area to develop a new treatment option [4]. In Rimpilä's study, PtcCO_2_ patterns were examined during several kinds of SDB, including persistent upper airway obstruction [5]. Sebastian describes that during hyperpnea, the snore signal can reveal where the upper airway collapses most frequently. It is therefore possible to use the snoring sound signal recording during sleep to detect the main location of the obstruction and improve treatment selection and outcomes [6]. Sawyer et al. describe that as it is agreeable to participants and can be applied effectively, clinical sleep centers are a suitable match for a personalized intervention method [7]. Berger et al. investigate whether intranasal leptin may alleviate obese hypoventilation and obstruction in upper airway in mice with DIO during sleep [8]. Lal et al. show that as a result of commercially accessible treatment options for OSA EDS, there has been improvement in different EDS indicators, as well as quality of life and job performance measurements [9]. Sharif et al. [10] proposed and used a novel procedure for work extraction from EEG. The calculation starts by building an implanting space utilizing EEG information. The calculation's affectability and low bogus expectation rate, for seizure forecast, showed its viability. The components used by Truong et.al. [11] are then standardized across the entire frequency spectrum to avoid high-frequency features from low-frequency features. Nolte et.al. [12] presented that Cartesian representation is better for examining brain connections because the typical magnitude and step of coherency involve the exact details as the actual and imagined sections. Mormann et.al. [13] presented that distinct shifts in spatial and temporal synchronization are sometimes related to pathological conduct. These measurements were used in this method to measure EEG recordings' phase synchronization after checking its robustness for noisy time series. Stam et.al. [14] presented electroencephalograms (EEG) and magnetoencephalograms (MEG) are two typical instances, each of which can require the simultaneous recording of 150 or more time series. Changes in alpha band synchronization, which are inseparable from eye-conclusion and enlightening, are a notable illustration of this marvel. Montazeri Ghahjaverestan [15] investigated the sleep apnea severity estimation, as the apnea/hypopnea index (AHI) was quantified, but the tidal volume estimated and extracted snoring sounds from signals of trachea. Tsao, C. H., et.al established the upper airway presence by renovating the changed sensory and motor function by vibration of hypoxia or snore. The flavor disorder (FD) risk is associated with OSA. In [16], the problem identification dealt with community-based research has demonstrated that sleep apnea is linked to various cardiovascular events, including coronary heart disease. For the SHHS OSA population, we first look at baseline symptoms to see whether any of the previously defined clinical categories present.

### 2.1. Proposed Methodology

Neurological issues with distinctive sorts of disorders are continuously happing, that is, ventilation on heart failure patients with sleep apnea snore, a persistent neurodegenerative infection that ordinarily begins one small step and develops over the long run. Heart failures are often considered hopeless, with never-ending heart issues that slowly harm body parts and affect the capacity of all organs to proceed with their fundamental assignments. This indication initially shows up in their heart-60s. Yet, presently it happened in the 50s-40s, and it will be more important to recognize this failure in starting phase as a piece of medical services with the support of ECG signal dissecting associated potentials (ERPs) blend with multirole arrangement wavelet investigation of Daubechies and Eyelets Grouping Recurrence groups that utilise AdaBoost and Multilayer Peception based decisions on medical ventilation for heart failure patients [17–19].

A brief description of cardiac disorders and the diagnostic procedure is provided in this article; in recent years, deep learning models have become increasingly popular for identifying any pattern or computed tomographs. The older models are helpful, but the location and influencing region are difficult to categorize. Existing models can detect neurological defects, Down syndrome, and congenital cardiac problems. To overcome the aforementioned restrictions, a powerful LeNet 6 deep learning classifier is required. The workflow comprises of image selection (CTA/ultrasound/fetal magnetic resonance), and image preprocessing procedures in the second stage are used to obtain an image with a high perceptual visual quality. In the third stage, OStU segmentation is used to extract features from the input heart picture. For illness localization and impacted region categorization, a final training and testing procedure is used. Finally, the proposed model diagram is shown in Figure 2.

In this work, at first-stage heart failure dataset is applied, in the next stage .csv file is filtered using auto stack encoder. The ventilation issues are used to extract features, after that classification is performed through LeNet-100 architecture [20–22].

#### 2.1.1. LeNet-100 Model

(1) $$\begin{array}{c} CWT_{n}\left(s,b\right)=\frac{1}{\sqrt{s}}\sum_{n=1}^{N-1}x\left(n\right)\Psi *\left(\frac{n-b}{s}\right). \end{array}$$

Time inhibitions of apparition parts might be procured by multiassurance CNN assessment, as this system offers a time-repeat depiction of the banner. The “LeNet-100” is used, and it can deal with an alternate course of action of issues, including data pressure, biomedical examination, feature extraction, clatter covering, work speculation, and thickness assessment, all with modest computational cost.

The LeNet-100 described as the difficulty of banner x(t) through wavelet limits *ψ*a,b(t), here *ψ*a,b(t) be enlarged and stimulated interpretation of wavelet work *ψ*(t) and is portrayed as takes after as mentioned in the following equation :

(2) $$\begin{array}{c} \Psi_{a,b}\left(t\right)=\sqrt{a.}\Psi \left(\frac{t-b}{a}\right). \end{array}$$

Autonomous parameters, that is, *a* and *b* in this technique, are excessive and not capable of methodological implementations as given in the following equation:

(3) $$\begin{array}{c} a_{j}=2^{-j},\;\\ b_{j,k}=2^{-j}.k\left(j,k\text{are integers}\right). \end{array}$$

In the LeNet-100 isolates, the banner disintegrates into several distinct recurrent packs. The high- and low-pass channels are utilized as a part of LeNet-100 that provides two courses of action: limits, scaling cutoff, Φ(t), and wavelet work, *ψ*(t), are given as follows:

(4) $$\begin{array}{c} \phi \left(t\right)=\sum_{n}h\left[n\right]\phi \left(2t-n\right), \end{array}$$

(5) $$\begin{array}{c} \Psi \left(t\right)=\sum_{n}g\left[n\right]\Psi \left(2t-n\right). \end{array}$$

On the other side, a wavelet work Ψ_*j*,*k*_(*t*) or scaling limit *ϕ*_*j*,*k*_(*t*) that will be discretized at level *j* and conversion *k* might exist procured as of principal work *ψ*(t) = *ψ*0, 0(t) or Φ (*t*) = Φ 0, 0(t), which are as follows:

(6) $$\begin{array}{c} \phi_{j,k}\left(t\right)=2^{-j/2}\phi \left(2^{-j}t-k\;\right), \end{array}$$

(7) $$\begin{array}{c} \Psi_{j,k}\left(t\right)=2^{-j/2}\Psi \left(2^{-j}t-k\;\right). \end{array}$$

We can get exact repeat and time limits of the banner using various scales and translations of these limits. The h(n) and g(n) coefficients (loads) accomplish the circumstances of 2.2 and 2.3 are the inspiration responses of low-pass and high-pass bands used in wavelet analysis, respectively, and characterize a wavelet used in the study. The flag decay into different repeat bunches is refined by reformist high-pass and low-take region signal.

To the degree of systematized accurate rehash, the most astonishing repeat in primary pennant is *π*, diverging from the prompt recurrence of 128 Hz. As indicated by Nyquist's manage, the colossal piece of the preceeding takes over after this process as mentioned in the following equations:

(8) $$\begin{array}{c} d_{1\;}\left[k\right]=y_{\text{high }}\left[k\right]\;=\sum_{n\;}x\left[n\right].g\left[2k-n\right], \end{array}$$

(9) $$\begin{array}{c} a_{1\;}\left[k\right]=y_{\text{low}}\left[k\right]=\sum_{n}x\left[n\right].h\left[2k-n\right]. \end{array}$$

This system either requires numerous comparative times for debilitating, or there will be more subsampling pending that is conceivable. On every stage, the structure accomplishes a limited quantity of point affirmation (taking into account subsampling) and are folded twice for recurrent confirmation (considering secluding), engaging the standard to be analyzed at various recurrent reaches within the wake of subsampling as mentioned the below equations;

(10) $$\begin{array}{c} A_{1}\left(t\right)=\sum_{k}a_{j}\left[k\right].\phi_{j,k}\left(t\right), \end{array}$$

(11) $$\begin{array}{c} D_{j}\left(t\right)=\sum_{k}d_{j}\left[k\right].\Psi_{j,k}\left(t\right), \end{array}$$

(12) $$\begin{array}{c} x\left(t\right)=A_{j}\left(t\right)+\overset{j}{\underset{j=-\infty }{\sum }}D_{j}\left(t\right)=\sum_{k}a_{j}\left(k\right).\phi_{j,k}\left(t\right)+\overset{j}{\underset{j=-\infty }{\sum }}\sum_{k}d_{j}\left[k\right].\Psi_{j,k}\left(t\right). \end{array}$$

Table 1 clearly explains about different samples, that is the following 14 attributes were used: 1. #3 (age); 2. #4 (sex); 3. #9 (cp); 4. #10 (trestbps); 5. #12 (chol); 6. #16 (fbs); 7. #19 (restecg); 8. #32 (thalach); 9. #38 (exang); 10. #40 (oldpeak); 11. #41 (slope); 12. #44 (ca); 13. #51 (thal); and 14. #58 (num) (the predicted attribute) target parameters taken.

## 3. Results and Discussion

This section discusses heart ventilation failure images and corresponding csv samples. These samples retrieve data from auto stack encoder, which is shown in Figure 3.

Figures 4 and 5 show the input heart picture, which is used to feed data into our proposed model after they have been segmented. The disease-affected region may be seen in this segmented picture.

In Figure 6, the darker color region clearly illustrates that the location of illness is primarily influenced by disease. Here, the features of the input image have been extracted using LeNet-10 CNN modeling.

Figure 7 clearly describes the GUI model of the suggested work. The input from the dataset has been implemented using the uploading function. The following action is granting access to segmentation module, which is shown in Table 2.

Figure 8 describes comparison of deep stacked, AGWO, and LeNet-100, and Table 3 represents the estimation of performance metrics for AdaBoost, OGP MLP OGP, specificity, sensitivity, NPV, and PPV.

Figure 9 shows the comparison of ECG analysis, and Table 4 represents the comparison results for various techniques like NB + KNN, nonlinear multidomain, deep stacked, AWGO deep stacked, WDS + ENR model, and proposed BP-ASE and LeNet-100.

Figure 10 shows the results of comparison; it is observed that the proposed method achieves accuracy, specificity, and sensitivity of 99.396, 95.38, and 99.12, respectively for training data, and for K-fold data, they are 99.41, 96.12, and 97.13, respectively.

## 4. Conclusion

When there is a problem with ventilation in the heart, it might lead to death. The apnea-hypopnea index (AHI) has historically been influenced by medical ventilation on heart failure; nevertheless, the sleep snore analysis is the best model to diagnose. The problems with ventilation are caused by problems with air pressure and blood circulation in the heart valves, where the pathological measurements are constantly identifying difficulties with ventilation. Understanding the pathogenesis of OSA will have a direct influence on clinical treatment decisions and clinical trial design. Signs and results of OSA therapy might be better understood by patients and researchers. Researchers may be able to determine which patient populations would most benefit from different OSA treatment options. To get information and apply classification algorithms, a LeNet-100 CNN-based deep learning technology is employed in this study. This performing meta-analysis obtained the heart failure dataset from the Kaggle website. An accuracy of 93.25 percent, sensitivity of 97.29 percent, recall of 96.34 percent, and F measure of 95.34 percent were all achieved. This approach outperforms technology and is comparable to current heart failure meta-analysis. In future, this work is enhanced by latest fine-grained algorithms for improving the efficiency of the system by considering huge data volume.

## Figures and Tables

**Figure 1:** Heart failure due to different effects.

**Figure 2:** Proposed model block diagram.

**Figure 3:** Heart ventilation issues.

**Figure 4:** Filtered image.

**Figure 5:** Disease location.

**Figure 6:** Gui model of proposed design.

**Figure 7:** Disease detection area.

**Figure 8:** Comparison of deep stacked, AGWO, and LeNet-100.

**Figure 9:** Comparison of ECG analysis.

**Figure 10:** Results of comparison.

**Table 1:** Dataset.

Age	Sex	CP	Trestbps	Chol	FBS	Rest ECG	Thalach	Exang	Oldpeak	Slope	CA	Thal	Target
52	1	0	125	212	0	1	168	0	1	2	2	3	0
53	1	0	140	203	1	0	155	1	3.1	0	0	3	0
70	1	0	145	174	0	1	125	1	2.6	0	0	3	0
61	1	0	148	203	0	1	161	0	0	2	1	3	0
62	0	0	138	294	1	1	106	0	1.9	1	3	2	0
58	0	0	100	248	0	0	122	0	1	1	0	2	1
58	1	0	114	318	0	2	140	0	4.4	0	3	1	0
55	1	0	160	289	0	0	145	1	0.8	1	1	3	0
46	1	0	120	249	0	0	144	0	0.8	2	0	3	0
54	1	0	122	286	0	0	116	1	3.2	1	2	2	0
71	0	0	112	149	0	1	125	0	1.6	1	0	2	1
43	0	0	132	341	1	0	136	1	3	1	0	3	0
34	0	1	118	210	0	1	192	0	0.7	2	0	2	1
51	1	0	140	298	0	1	122	1	4.2	1	3	3	0
52	1	0	128	204	1	1	156	1	1	1	0	0	0
34	0	1	118	210	0	1	192	0	0.7	2	0	2	1
51	0	2	140	308	0	0	142	0	1.5	2	1	2	1
54	1	0	124	266	0	0	109	1	2.2	1	1	3	0
50	0	1	120	244	0	1	162	0	1.1	2	0	2	1
58	1	2	140	211	1	0	165	0	0	2	0	2	1
60	1	2	140	185	0	0	155	0	3	1	0	2	0
67	0	0	106	223	0	1	142	0	0.3	2	2	2	1
45	1	0	104	208	0	0	148	1	3	1	0	2	1
63	0	2	135	252	0	0	172	0	0	2	0	2	1
42	0	2	120	209	0	1	173	0	0	1	0	2	1
61	0	0	145	307	0	0	146	1	1	1	0	3	0
44	1	2	130	233	0	1	179	1	0.4	2	0	2	1
58	0	1	136	319	1	0	152	0	0	2	2	2	0
56	1	2	130	256	1	0	142	1	0.6	1	1	1	0
55	0	0	180	327	0	2	117	1	3.4	1	0	2	0
44	1	0	120	169	0	1	144	1	2.8	0	0	1	0
50	0	1	120	244	0	1	162	0	1.1	2	0	2	1
57	1	0	130	131	0	1	115	1	1.2	1	1	3	0
70	1	2	160	269	0	1	112	1	2.9	1	1	3	0
50	1	2	129	196	0	1	163	0	0	2	0	2	1
46	1	2	150	231	0	1	147	0	3.6	1	0	2	0
51	1	3	125	213	0	0	125	1	1.4	2	1	2	1
59	1	0	138	271	0	0	182	0	0	2	0	2	1
64	1	0	128	263	0	1	105	1	0.2	1	1	3	1
57	1	2	128	229	0	0	150	0	0.4	1	1	3	0
65	0	2	160	360	0	0	151	0	0.8	2	0	2	1
54	1	2	120	258	0	0	147	0	0.4	1	0	3	1
61	0	0	130	330	0	0	169	0	0	2	0	2	0
46	1	0	120	249	0	0	144	0	0.8	2	0	3	0
55	0	1	132	342	0	1	166	0	1.2	2	0	2	1
42	1	0	140	226	0	1	178	0	0	2	0	2	1
41	1	1	135	203	0	1	132	0	0	1	0	1	1
66	0	0	178	228	1	1	165	1	1	1	2	3	0
66	0	2	146	278	0	0	152	0	0	1	1	2	1
60	1	0	117	230	1	1	160	1	1.4	2	2	3	0
58	0	3	150	283	1	0	162	0	1	2	0	2	1
57	0	0	140	241	0	1	123	1	0.2	1	0	3	0
38	1	2	138	175	0	1	173	0	0	2	4	2	1
49	1	2	120	188	0	1	139	0	2	1	3	3	0
55	1	0	140	217	0	1	111	1	5.6	0	0	3	0
55	1	0	140	217	0	1	111	1	5.6	0	0	3	0
56	1	3	120	193	0	0	162	0	1.9	1	0	3	1
48	1	1	130	245	0	0	180	0	0.2	1	0	2	1
67	1	2	152	212	0	0	150	0	0.8	1	0	3	0
57	1	1	154	232	0	0	164	0	0	2	1	2	0
29	1	1	130	204	0	0	202	0	0	2	0	2	1
66	0	2	146	278	0	0	152	0	0	1	1	2	1
67	1	0	100	299	0	0	125	1	0.9	1	2	2	0
59	1	2	150	212	1	1	157	0	1.6	2	0	2	1
29	1	1	130	204	0	0	202	0	0	2	0	2	1
59	1	3	170	288	0	0	159	0	0.2	1	0	3	0
53	1	2	130	197	1	0	152	0	1.2	0	0	2	1
42	1	0	136	315	0	1	125	1	1.8	1	0	1	0
37	0	2	120	215	0	1	170	0	0	2	0	2	1
62	0	0	160	164	0	0	145	0	6.2	0	3	3	0
59	1	0	170	326	0	0	140	1	3.4	0	0	3	0
61	1	0	140	207	0	0	138	1	1.9	2	1	3	0
56	1	0	125	249	1	0	144	1	1.2	1	1	2	0
59	1	0	140	177	0	1	162	1	0	2	1	3	0
48	1	0	130	256	1	0	150	1	0	2	2	3	0
47	1	2	138	257	0	0	156	0	0	2	0	2	1
48	1	2	124	255	1	1	175	0	0	2	2	2	1
63	1	0	140	187	0	0	144	1	4	2	2	3	0
52	1	1	134	201	0	1	158	0	0.8	2	1	2	1
52	1	1	134	201	0	1	158	0	0.8	2	1	2	1
50	1	2	140	233	0	1	163	0	0.6	1	1	3	0
49	1	2	118	149	0	0	126	0	0.8	2	3	2	0
46	1	2	150	231	0	1	147	0	3.6	1	0	2	0
38	1	2	138	175	0	1	173	0	0	2	4	2	1
37	0	2	120	215	0	1	170	0	0	2	0	2	1
44	1	1	120	220	0	1	170	0	0	2	0	2	1
58	1	2	140	211	1	0	165	0	0	2	0	2	1
59	0	0	174	249	0	1	143	1	0	1	0	2	0
62	0	0	140	268	0	0	160	0	3.6	0	2	2	0
68	1	0	144	193	1	1	141	0	3.4	1	2	3	0
54	0	2	108	267	0	0	167	0	0	2	0	2	1
62	0	0	124	209	0	1	163	0	0	2	0	2	1
63	1	0	140	187	0	0	144	1	4	2	2	3	0
44	1	0	120	169	0	1	144	1	2.8	0	0	1	0
62	1	1	128	208	1	0	140	0	0	2	0	2	1
45	0	0	138	236	0	0	152	1	0.2	1	0	2	1
57	0	0	128	303	0	0	159	0	0	2	1	2	1
53	1	0	123	282	0	1	95	1	2	1	2	3	0
65	1	0	110	248	0	0	158	0	0.6	2	2	1	0

**Table 2:** Comparison of results.

Parameter	Deep stacked	AGWO	LeNet-100
True positive rate	0.872	0.912	0.943
F1 score	0.893	0.934	0.951
MNSE	0.062	0.04	0.01

**Table 3:** Estimation of performance metrics.

Sym5	AdaBoost OGP	MLP OGP	Specificity	Sensitivity	NPV	PPV
TFz2–4 Hz	55.8	54.7	57.5	60.7	55.6	62.6
TCz2–4 Hz	53.8	53.0	55.8	51.4	49.5	57.8
TPz2–4 Hz	51.3	50.6	41.7	47.1	40.1	48.6
NCz2–4 Hz	64.1	63.2	60.0	58.6	55.0	63.6
NPz 2-4 Hz	**87.8**	**84.2**	**98.3**	**98.5**	**98.6**	**98.4**
NFz2–4 Hz	54.5	53.6	52.5	47.9	46.4	53.9

**Table 4:** Comparison of results.

Models		NB + KNN	Nonlinear multidomain	Deep stacked	AWGO deep stacked	WDS + ENR model	BP-ASE and LeNet-100
Training data	Accuracy	87.9623	91.9692	92.6	94.1035	98.78	99.396
	Specificity	88.8321	91.243	91.8	91.9832	92.32	95.38
	Sensitivity	58.6483	84.41	97.22	97.3456	98.52	99.12
K-fold data	Accuracy	92.1374	93.26	93.45	93.6431	97.732	99.41
	Specificity	91.2389	91.56	91.8	91.984	95.74	96.12
	Sensitivity	92.6552	92.8	92.3	93	96.94	97.13

## Data Availability

No data were used to support this study.

## References

[1] Edwards B. A., Redline S., Sands S. A., Owens R. L. (2019). More than the sum of the respiratory events: personalized medicine approaches for obstructive sleep apnea. *American Journal of Respiratory and Critical Care Medicine*.

[2] Coleman J. M., Wolfe L. F., Kalhan R. (2019). Noninvasive ventilation in chronic obstructive pulmonary disease. *Annals of the American Thoracic Society*.

[3] Kersin B., Karaman M., Aynacı E., Keleş A. (2020). Investigation of the effectiveness of surgical treatment on respiratory functions in patients with obstructive sleep apnea syndrome. *Ear, Nose, & Throat Journal*.

[4] Carter T. (2020). Mandibular attachment device effects on African American veterans with heart failure.

[5] Sampathkumar A., Murugan S., Rastogi R., Mishra M. K., Malathy S., Manikandan R. (2020). Energy efficient ACPI and JEHDO mechanism for IoT device energy management in healthcare. *Internet of Things in Smart Technologies for Sustainable Urban Development*.

[6] Sebastian A. (2021). Identifying the site of upper airway collapse in obstructive sleep apnoea patients using snore signals.

[7] Sawyer A. M., King T. S., Weaver T. E. (2019). A tailored intervention for PAP adherence: the SCIP-PA Trial. *Behavioral Sleep Medicine*.

[8] Berger S., Pho H., Fleury-Curado T. (2019). Intranasal leptin relieves sleep-disordered breathing in mice with diet-induced obesity. *American Journal of Respiratory and Critical Care Medicine*.

[9] Lal C., Weaver T. E., Bae C. J., Strohl K. P. (2021). Excessive daytime sleepiness in obstructive sleep apnea. Mechanisms and clinical management. *Annals of the American Thoracic Society*.

[10] Sobral D. S., Faller G. J., Collares M. V. M. (2018). Respiratory polysomnographic findings in patients treated primarily for unilateral cleft lip and palate. *The Cleft Palate-Craniofacial Journal*.

[11] Jensen H. (2017). *Primary Care Strategies for the Screening of Obstructive Sleep Apnea in Children: An Integrative Review*.

[12] Ramesh S., Nirmalraj S., Murugan S., Manikandan R., Al-Turjman F. (2021). Optimization of energy and security in mobile sensor network using classification based signal processing in heterogeneous network. *Journal of Signal Processing Systems*.

[13] Bianchi A. M., Villantieri O. P., Mendez M. O., Patruno V., Cerutti S., Montano N. Different effects of CPAP and APAP therapies on the autonomic nervous system in OSA patients.

[14] Hsia J. C. (2015). Anatomy and physiology of the upper airway in obstructive sleep apnea. *Operative Techniques in Otolaryngology - Head and Neck Surgery*.

[15] MontazeriGhahjaverestan N., Saha S., Kabir M., Gavrilovic B., Zhu K., Yadollahi A. (2021). Sleep apnea severity based on estimated tidal volume and snoring features from tracheal signals. *Journal of Sleep Research*.

[16] Chien-Han T., Huang J., Huang H., Hung Y., Wei J. C., Tsan H. Y. (2019). Ankylosing spondylitis is associated with risk of new onset obstructive sleep apnea: a nationwide population-based cohort study. *Frontiers in Medicine*.

[17] Hoon K., Jong H. K., Kyung-jin A. (2020). Smart home energy strategy based on human behaviour patterns for transformative computing. *Information Processing & Management*.

[18] Kim M. G., Ko H., Pan S. B. (2019). A study on user recognition using 2D ECG based on ensemble of deep convolutional neural networks. *Journal of Ambient Intelligence and Humanized Computing*.

[19] Ko H., Pan S. B., Mesicek L. (2020). Personal identification study for touchable devices with ECG. *Concurrency and Computation: Practice and Experience*.

[20] Lv Z., Ko H. (2021). Introduction to the special issue on recent trends in medical data security for e-health applications. *ACM Transactions on Multimedia Computing, Communications, and Applications*.

[21] Elhoseny M., Ramírez-González G., Abu-Elnasr O. M., Shawkat S. A., Arunkumar N., Farouk A. (2018). Secure medical data transmission model for IoT-based healthcare systems. *Ieee Access*.

[22] Abdolmaleky M., Naseri M., Batle J., Farouk A., Gong L. H. (2017). Red-Green-Blue multi-channel quantum representation of digital images. *Optik*.

